# Water Quality Prediction Using Artificial Intelligence Algorithms

**DOI:** 10.1155/2020/6659314

**Published:** 2020-12-29

**Authors:** Theyazn H. H Aldhyani, Mohammed Al-Yaari, Hasan Alkahtani, Mashael Maashi

**Affiliations:** ^1^Community College of Abqaiq, King Faisal University, P.O. Box 400, Al-Ahsa 31982, Saudi Arabia; ^2^Chemical Engineering Department, King Faisal University, P.O. Box 380, Al-Ahsa 31982, Saudi Arabia; ^3^College of Computer Science and Information Technology, King Faisal University, P.O. Box 400, Al-Ahsa 31982, Saudi Arabia; ^4^Software Engineering Department, King Saud University, Riyadh 11543, Saudi Arabia

## Abstract

During the last years, water quality has been threatened by various pollutants. Therefore, modeling and predicting water quality have become very important in controlling water pollution. In this work, advanced artificial intelligence (AI) algorithms are developed to predict water quality index (WQI) and water quality classification (WQC). For the WQI prediction, artificial neural network models, namely nonlinear autoregressive neural network (NARNET) and long short-term memory (LSTM) deep learning algorithm, have been developed. In addition, three machine learning algorithms, namely, support vector machine (SVM), *K*-nearest neighbor (K-NN), and Naive Bayes, have been used for the WQC forecasting. The used dataset has 7 significant parameters, and the developed models were evaluated based on some statistical parameters. The results revealed that the proposed models can accurately predict WQI and classify the water quality according to superior robustness. Prediction results demonstrated that the NARNET model performed slightly better than the LSTM for the prediction of the WQI values and the SVM algorithm has achieved the highest accuracy (97.01%) for the WQC prediction. Furthermore, the NARNET and LSTM models have achieved similar accuracy for the testing phase with a slight difference in the regression coefficient (RNARNET = 96.17% and RLSTM = 94.21%). This kind of promising research can contribute significantly to water management.

## 1. Introduction

Water is the most significant resource of life, crucial for supporting the life of most existing creatures and human beings. Living organisms need water with enough quality to continue their lives. There are certain limits of pollutions that water species can tolerate. Exceeding these limits affects the existence of these creatures and threatens their lives.

Most ambient water bodies such as rivers, lakes, and streams have specific quality standards that indicate their quality. Moreover, water specifications for other applications/usages possess their standards. For example, irrigation water must be neither too saline nor contain toxic materials that can be transferred to plants or soil and thus destroying the ecosystems. Water quality for industrial uses also requires different properties based on the specific industrial processes. Some of the low-priced resources of fresh water, such as ground and surface water, are natural water resources. However, such resources can be polluted by human/industrial activities and other natural processes.

Hence, rapid industrial development has prompted the decay of water quality at a disturbing rate. Furthermore, infrastructures, with the absence of public awareness, and less hygienic qualities, significantly affect the quality of drinking water [1]. In fact, the consequences of polluted drinking water are so dangerous and can badly affect health, the environment, and infrastructures. As per the United Nations (UN) report, about 1.5 million people die each year because of contaminated water-driven diseases. In developing countries, it is announced that 80% of health problems are caused by contaminated water. Five million deaths and 2.5 billion illnesses are reported annually [2]. Such a mortality rate is higher than deaths resulting from accidents, crimes, and terrorist attacks [3].

Therefore, it is very important to suggest new approaches to analyze and, if possible, to predict the water quality (WQ). It is recommended to consider the temporal dimension for forecasting the WQ patterns to ensure the monitoring of the seasonal change of the WQ [4]. However, using a special variation of models together to predict the WQ grants better results than using a single model [5–7]. There are several methodologies proposed for the prediction and modeling of the WQ. These methodologies include statistical approaches, visual modeling, analyzing algorithms, and predictive algorithms. For the sake of the determination of the correlation and relationship among different water quality parameters, multivariate statistical techniques have been employed [4]. The geostatistical approaches were used for transitional probability, multivariate interpolation, and regression analysis [5].

Massive increases in population, the industrial revolution, and the use of fertilizers and pesticides have led to serious effects on the WQ environments [8, 9]. Thus, having models for the prediction of the WQ is of great help for monitoring water contamination.

Currently, two main types for modeling and predicting water quality are available: mechanism- and non-mechanism-oriented models. The mechanism model is relatively sophisticated; it uses the advanced system structure data for simulating the WQ, and thus, it is considered as a multifunctional model that can be used for any water body. In addition, the Streeter–Phelos (S–P) model, one of the earliest WQ simulation model, has been used widely.

Later, some countries have developed a variety of WQ models including the QUAL model [10] and the WASP model [11], which have gained wide usage in mimicking the water quality of rivers. This was followed by Warren and Bach [12] who suggested to use MIKE21 for designing systems to model the estuaries, coastal waters, and seas.

Hayes et al. [13] have paired two models for improving the quality of downstream water, namely, quasi-static two-dimensional dissolved oxygen reservoir model (DORM-II) and a daily scale optimal dispatch model.

Using environmental fluid dynamics code (EFDC), a two-dimensional numerical model was developed to simulate the water environment of the Mudan River [14]. This is based on the distance between points and intervals [15].

Another study was conducted by Batur and Maktav [16] to predict the WQ of Lake Gala (Turkey) using satellite image fusion based on the principal component analysis (PCA) method. Jaloree et al. [17] have attempted to predict the WQ of the Narmada River with five WQ indicators using a decision tree model. Another study suggested the use of the deep Bidirectional Stacked Simple Recurrent Unit (Bi-S-SRU) [18] for the designing of a precise forecasting scheme of the WQ in smart mariculture.

Liao and Sun [19] developed a model to forecast the WQ of China's Chao Lake by pairing the ANN and decision tree algorithm. Yan and Qian [20] proposed an affinity propagation clustering model based on a least-squares support vector machine (AP-LSSVM). This model is highly sensitive to vacancies. Solanki et al. [21] analyzed and predicted the chemical eigenvalues of water, especially dissolved oxygen and pH using the deep learning network model which was reported to demonstrate more accurate results compared with supervised learning-based techniques. Li et al. [22] developed a novel hybrid model using a neural network and the Markov chain method. This model has helped in predicting dissolved oxygen, a primary measure of the WQ [23]. Khan and See [24] included dissolved oxygen, chlorophyll, conductivity, and turbidity in the developed WQ model using an artificial neural network (ANN). Yan et al. [25] suggested a genetic algorithm (GA) and particle swarm optimization (PSO) algorithm to enhance the backpropagation (BP) neural network to predict the oxygen demanded in a lake. An enhanced accuracy of the prediction results was reported.

Several studies have been performed to model and predict the water quality using different ANN models. These studies have approved the feasibility and effectiveness of employing ANN applications to predict the quality of drinking water.

Currently, researchers mostly emphasize enhancing the applicability and reliability of water quality prediction/modelling by using a variety of new technologies such as Fuzzy logic, stochastic, ANN, and deep learning [26, 27].

Shafi et al. [28] proposed four machine learning algorithms, namely, Support Vector Machines (SVM), Neural Networks (NN), Deep Neural Networks, and *k*-Nearest Neighbors (kNN), for the prediction of water quality. Using single feed-forward neural networks to classify water quality, 25 parameters have been included as input parameters [29].

Ranković et al. [30] estimated the dissolved oxygen (DO) by employing the ANN model. Gazzaz et al. [31] estimated the WQI by using an ANN model, and the Internet of Things (IOT) technology was applied to collect the dataset from water resources. Abyaneh [32] has applied the machine learning approaches like ANN and regression to predict the chemical oxygen demand (COD). Sakizadeh [33] used ANN with Bayesian regularization to estimate the water quality index (WQI). However, the radial-basis-function (RBF), a type of the ANN model, was used for the prediction and classification of water quality [34, 35].

In addition, it has been reported that deep learning methods showed high performance in predicting the WQ when compared to the traditional methods. Marir et al. [36] developed a model to find out the uncommon behavior from large-scale network traffic data. While a deep learning algorithm was employed for extracting features, a multilayer ensemble support vector machine model was used for classification. Fadlullah et al. [37] visualized a reward-based deep learning structure combining a deep convolutional neural network and a deep belief network.

For the analysis and prediction of the WQ of groundwater, different algorithms including ANN, Bayesian neural networks, adaptive neurofuzzy [38], decision support system (DSS), and autoregressive moving average (ARMA) have been applied [39]. However, these mimicking models have some limitations.

However, the contributions of the current study can be summarized as follows:

- Developing highly efficient advanced artificial intelligence models to predict the water quality index (WQI) based on artificial neural networks and deep learning algorithms
- Applying some machine learning models, namely, support vector machine (SVM), *K*-nearest neighbour (K-NN), and Naive Bayes algorithms, for the prediction of water quality classification (WQC).

The highly efficient developed models can be generalized and used to forecast the water pollution process which will help the decision-makers to make the right decisions at the right time.

## 2. Materials and Methods

Figure 1 displays the proposed methodology of the present study.

### 2.1. Dataset

The dataset used in this study is collected from certain historical locations in India. It contained 1679 samples from different Indian states during the period from 2005 to 2014. The dataset has 7 significant parameters, namely, dissolved oxygen (DO), pH, conductivity, biological oxygen demand (BOD), nitrate, fecal coliform, and total coliform. Data was collected by the Indian government to ensure the quality of the supplied drinking water. This dataset was obtained from Kaggle https://www.kaggle.com/anbarivan/indian-water-quality-data.

### 2.2. Data Preprocessing

The processing phase is very important in data analysis to improve the data quality. In this phase, the WQI has been calculated from the most significant parameters of the dataset. Then, water samples have been classified on the basis of the WQI values. For obtaining superior accuracy, the *z*-score method has been used as a data normalization technique.

#### 2.2.1. Water Quality Index Calculation

To measure water quality, WQI is used to be calculated using various parameters that significantly affect WQ [40–42]. In this study, a published dataset is considered to test the proposed model, and seven significant water quality parameters are included. The WQI has been calculated using the following formula:

(1) $$\begin{array}{c} \text{WQI}=\frac{\sum_{i=1}^{N}q_{i}\times w_{i}}{\sum_{i=1}^{N}w_{i}}, \end{array}$$

where: *N* is the total number of parameters included in the WQI calculations*q*_*i*_ is the quality rating scale for each parameter *i* calculated by equation (2) below, and *w*_*i*_ is the unit weight for each parameter calculated by equation (3).

(2) $$\begin{array}{c} q_{i}=100\times \left(\frac{V_{i}-V_{\text{Ideal}}}{S_{i}-V_{\text{Ideal}}}\right), \end{array}$$

where:*V*_*i*_ is the measured value of parameter *i* in the tested water samples*V*_Ideal_ is the ideal value of parameter *i* in pure water (0 for all parameters except DO = 14.6 mg/l and pH = 7.0), and *S*_*i*_ is the recommended standard value of parameter *i* (as shown in Table 1).

(3) $$\begin{array}{c} w_{i}=\frac{K}{S_{i}}, \end{array}$$

where *K* is the proportionality constant that can be calculated as follows:

(4) $$\begin{array}{c} \;K=\frac{1}{\sum_{i=1}^{N}S_{i}}, \end{array}$$

Tables 2 and 3 represent the unit weight of each parameter and the WQC, respectively.

#### 2.2.2. *Z*-Score Normalization Method

Normalization is a way to simplify calculations. It is a dimensional expression transformed into a nondimensional expression and becomes a scalar. *Z*-score normalization (or normalization score) is a normalization method used to normalize parameters by using the mean (*μ*) and standard deviation (*σ*) values of the tested data. It can be calculated as follows:

(5) $$\begin{array}{c} Z‐\text{score}=\frac{\left(x-\mu \right)}{\sigma }, \end{array}$$

where *x* is the measured value of the parameter *i* in the tested sample.

### 2.3. Prediction of Water Quality Index

For this purpose, ANN models, namely, nonlinear autoregressive neural network (NARNET) and long short-term memory (LSTM) deep learning algorithm, were used for the prediction of water quality index.

#### 2.3.1. Artificial Neural Network (ANN) Model

In general, the neural network (NN) models are used as very powerful machine learning algorithms for time-series prediction of different engineering applications. The ANN model has consisted of an input layer, a hidden layer/s, and an output layer. Each hidden layer has weight and bias parameters to manage neurons. To transfer the data from the hidden layer into the output layer, the activation function is used. The learning algorithms are used to select the weights within the NN framework. The weight selection is based on the minimum performance measures such as mean square error (MSE).

The NARNET model is a very popular multilayer feed-forward network. It starts with a guessed initial weight value, which is then updated using the actual data. Consequently, there is some sort of randomness in the prediction process performed by the NN model. The network is regularly trained many times using different random values for the initialization, and the results are averaged. In the NARNET model, the number of hidden layers and nodes must be identified in advance.  Figure 2 displays the NARNET model scheme with multiple inputs and 4 hidden layers (as recommended for most of the research datasets). Equation (6) describes the NARNET time series model.

(6) $$\begin{array}{c} y\left(t\right)=h\left(y\left(t-1\right),y\left(t-2\right),\cdots ,y\left(t-p\right)\right)+\epsilon \left(t\right), \end{array}$$

where *y* is the value of time-series data at time *t* and *y*(*t*) for employing the *p* observation values of the series. The function (*h*) is used to optimize the network weights and neuron bias. Finally, the *ϵ*(*t*) is the error obtained from the model at time *t*.

In this work, the NARNET model has been developed to predict the WQI. The NARNET model is a time series model that is used to predict the stationary time series compared with other ANN models like the forward neural network model. The WQI parameters seem in the form of time series; therefore, the NARNET model is proposed to predict the WQI.  Table 4 shows the significant parameters of the developed model.  Figure 3 represents the topology of the developed NARNET model.

#### 2.3.2. Deep Neural Network (DNN) Model

The DNN model is one type of feedforward NN algorithms, which is a fundamental technique for deep learning. DNN consists of 3 levels of nodes, and each node follows a nonlinear function, except for the input node. DNN presents a technique of backpropagation supervised learning. In this work, a WQI model was developed using the DNN algorithm and the simple DNN was compared with the proposed model. This model includes the following parameters and functions: bias (*b*), input (*x*), output (*y*), weight (*w*), calculation function (*α*), and activation function *f*(*α*). The neuron architecture of the DNN model is schematically shown in Figures 4and 5. Every single neuron in the DNN employs the following equations.

(7) $$\begin{array}{c} \alpha :sum=w∙x+b, \end{array}$$

(8) $$\begin{array}{c} y:f\left(\alpha \right)=f\left(w∙x+b\;\right), \end{array}$$

Recurrent neural network (RNN) is one type of deep learning techniques used in different domains such as computer vision, natural language processing, pattern recognition, and medical image diagnosis. As compared to different feed ANNs, RNN has a directional control loop that enables the previous states to be stored, recalled, and added to the current output. One of the most powerful RNN algorithms used to predict time series data is the LSTM model.

The long short-term memory (LSTM) model, a deep learning algorithm, is appropriate for estimating the time-series data whenever there is a randomized sized time step. The activating function used in the LSTM model is a logistic sigmoid. Providing that the forget gate is opened and the input gate is closed, the memory cell keeps reminding of the first entry and thus solving the typical RNN problems [44]. The formulas of the RNN model are as follows:

(9) $$\begin{array}{c} h_{t}=\tan h\left(W_{i}∙h_{t}+w_{x}\;x_{t}\right), \end{array}$$

(10) $$\begin{array}{c} y_{t}=w_{y}∙w_{t}, \end{array}$$

where *h*_*t*_ is the hidden layer of NN for the input training data (*x*_*t*_). The output layer is represented by *y*_*t*_. However, *w*_*t*_ and *w*_*y*_ are the weight of the neural cell and the matrix, respectively. The RNN model is used to create the LSTM model for the computing process. The LSTM consists of three significant parameters, namely, the input gate, forget gate, and output gate. The formulas used to compute the LSTM model are as follows:

(11) $$\begin{array}{c} \text{Input gate}:i_{t}=\sigma \left(W_{i}∙\left[h_{t-1},x_{t}\right]+b_{i}\right), \end{array}$$

(12) $$\begin{array}{c} \text{Forget gate}:f_{t}=\sigma \left(w_{f}∙\left[h_{t-1},x_{t}\;\right]+b_{f}\right), \end{array}$$

(13) $$\begin{array}{c} \text{Output gate}:o_{t}=\sigma \left(W_{0}∙\left[h_{t-1},x_{t}\right]+b_{0}\right), \end{array}$$

(14) $$\begin{array}{c} \text{New memory cell}:{\tilde{c\;}}_{t}=\tan h\left(W_{c}∙\left[h_{t-1},x_{t}\;\right]+b_{c}\right), \end{array}$$

(15) $$\begin{array}{c} \text{Final memory cell}:C_{t}=f_{t}\times C_{t-1}+i_{t}\times {\tilde{\;c\;}}_{t}, \end{array}$$

(16) $$\begin{array}{c} h_{t}=o_{t}\times \tan h\left(C_{t}\right), \end{array}$$

where:

*i*_*t*_, *f*_*t*_, and *o*_*t*_: input, forget, and output gates, respectively

 *h*_*t*_: number of hidden layers

*σ*: the logistic sigmoid function is used to transfer the training data from a hidden layer into the output gate

*w*_*t*_: the weighted neural network

${\tilde{\;c\;}}_{t}:$ an internal memory cell is used to compute in the hidden layer

*C*_*t*_: the internal memory

*h*_*t*_:the output of a hidden layer state is used to derive from the new memory

*i*, *f*, and *o*: are subscripts that stand for input, forget, and output gates, respectively

*x*_*t*_: input training data

*w*_*f*_, *w*_*o*_*w*_*c*_: weight vector of NN

*b*_*f*_ and *b*_*o*_: bias vector in NN

The analysis of LSTM was performed utilizing MATLAB. Throughout the LSTM layer, 23 variables are open. We just set the units, activate the function, return the sequence, and dropout.  Figure 5 illustrates the architecture of the LSTM, and the significant parameters of the LSTM model are presented in Table 5.

### 2.4. Prediction of Water Quality Classification

In this section, some machine learning algorithms, namely, support vector machine (SVM), *K*-nearest neighbor (KNN), and Naive Bayes, have been used to predict the water quality classification.

#### 2.4.1. Support Vector Machine (SVM) Model

The SVM model was developed in 1995 by Corinna Cortes and Vapnik. It has several unique benefits in solving small samples, and nonlinear and high-dimensional pattern recognition. It can be extended to function in the simulation of other machine learning problems. It uses the hyperplane to separate the points of the input vectors and finds the needed coefficients. The best hyperplane is the line with the largest margin, which is meant the distance between the hyperplane and the nearest input objects. The input points defined in the hyperplane are called *support vectors*. In this work, the linear SVM model along with the Gaussian radial basis function (equation (17)) is used to classify the tested water samples based on their quality.

(17) $$\begin{array}{c} K\left(X,X^{\prime }\right)=\exp\left(-\frac{{\left|\left|X-X^{\prime }\right|\right|}^{2}}{2\sigma^{2}}\right), \end{array}$$

where *X* and *X*′ represent the feature vectors of the input dataset and the ‖*X* − *X*′‖^2^ is the squared Euclidean distance between the two feature inputs. The *σ* is a free parameter.

#### 2.4.2. *K*-Nearest Neighbor (K-NN) Model

The K-NN algorithm is a basic classification and regression method. It is used to find the *K* values that are close to values in the training dataset. Most of these values belong to a certain class, and thus, tested data can be classified. The *K* value is used to find the closest points in the feature vectors, and the value should be unique. The following expression of the Euclidean distance function (Di) can be used.

(18) $$\begin{array}{c} D_{i}=\sqrt{\left(x_{1}-x_{2}\right)+{\left(y_{1}-y_{2}\right)}^{2},} \end{array}$$

where *x*_1_, *x*_2_, *y*_1_, and *y*_2_ are the variables for input data.

#### 2.4.3. Naive Bayes Model

The Bayesian method uses the knowledge of probability statistics to predict and classify datasets. The Bayesian algorithm combines prior and posterior probabilities to avoid the supervisor's bias and the overfitting phenomenon of using sample information alone.

This Naive Bayes is a type of classification algorithms based on Bayes' theorem and the assumption of the independence of characteristic conditions. Attributes are assumed to be conditionally independent of each other when the target value is given. This method greatly simplifies the complexity of the Bayesian method.

In Bayesian analysis, the probability of an event A given an event B is not the same as the probability of *B* given *A* as in equation (18).

(19) $$\begin{array}{c} P\left(A\;|\;B\right)\neq P\left(B\;|\;A\right). \end{array}$$

Assuming that *A*_1_, *A*_2_ ⋯ .*A*_*n*_ and *C* are the feature vectors and the class of the WQC dataset, respectively, the Bayes equation can be expressed as follows:

(20) $$\begin{array}{c} P\left(C\;|\;A\right)=\frac{P\left(C\right)\times P\left(A\;|\;C\right)}{P\left(A\right)}, \end{array}$$

where the *P*(*A*) is a prior probability representing the feature vectors of the WQC dataset and *P*(*A* | *C*) is the prior probability of the class of the WQC dataset.

### 2.5. Performance Measurement

The statistical analysis, namely, mean square error (MSE), has been used to evaluate the robustness of the developed models to predict the WQI. However, the accuracy, specificity, sensitivity, precision, and *F*-score evaluation matrices were employed to evaluate the developed classification model to predict the WQC. The used statistical parameters were defined as follows:

- Mean Square Error (MSE)

(21) $$\begin{array}{c} \text{MSE}=\frac{1}{N}\overset{N}{\underset{i=1}{\sum }}{\left(y_{i}-{\overset{\wedge }{y}}_{i}\right)}^{2}, \end{array}$$

where *y*_*i*_ and ${\hat{y}}_{i}$ are the predicted and the observed responses, respectively, and *N* is the total number of variables.

(b) Accuracy

(22) $$\begin{array}{c} \text{Accuracy}=\frac{\text{TP}+\text{TN}}{\text{TP}+\text{FP}+\text{FN}+\text{TN}}\times 100\%, \end{array}$$

(c) Specificity

(23) $$\begin{array}{c} \text{Specificity}=\frac{\text{TN}}{\text{TN}+\text{FP}}\times 100\%, \end{array}$$

(d) Sensitivity

(24) $$\begin{array}{c} \text{Sensitivity}=\frac{\text{TP}}{\text{TP}+\text{FN}}\times 100\%, \end{array}$$

(e) Precision

(25) $$\begin{array}{c} \text{Precision}=\frac{\text{TP}}{\text{TP}+\text{FP}}\times 100\%, \end{array}$$

(f) *F*-score

(26) $$\begin{array}{c} F‐\text{score}=\frac{2\times \text{precision}\times \text{sensitivity}}{preision+\text{sensitivity}}\times 100\%, \end{array}$$

where TP, TN, FP, and *FN* are the true positive, true negative, false positive, and false negative, respectively.

### 2.6. Correlation Analysis

Pearson's correlation coefficient approach is applied to analyze the correlation between the significant parameters of the dataset used for the prediction of the QWI values.

(27) $$\begin{array}{c} R=\frac{n\sum \left(x\times y\right)-\left(\Sigma x\right)\left(\Sigma y\right)}{\left[n\sum \left(x^{2}\right)-\sum \left(x^{2}\right)\right]\times \left[n\sum \left(y^{2}\right)-\sum \left(y^{2}\right)\right]}\times 100\%, \end{array}$$

where:

*R*: Pearson's correlation coefficient approach

*x*: input values in the first set of the training data

*y*: input values of the second set of the training data

*n*: total number of input variables

### 2.7. Experimental Setup

The prediction experiments have been conducted in a specific environment (MATLAB 2018). The simulation has been performed using a system with i5 Processor and 4 GB RAM to process all required tasks.

## 3. Results and Discussion

For validating the developed model, the dataset has been divided into 70% training and 30% testing subsets. While the ANN and LSTM models were used to predict the WQI, the SVM, KNN, and Naive Bayes were utilized for the water quality classification prediction.

### 3.1. Prediction of the WQI

A NARNET model, with 12 hidden layers, showed a good performance to predict the WQI values. As presented earlier, it has the following characteristics: 1 : 8 number of delays and 12 number of epochs. However, the developed LSTM model has a total number of 200 hidden layers,150 maximum number of epochs, and delays of [1, 3, 4, 7].

Table 6 summarizes the performance parameters of the developed models to predict WQI, although the prediction accuracy of LSTM for the testing data was slightly better than that for the training data. In addition, the LSTM model, in general, has shown a slightly better performance compared with the NARNET model according to the MSE values. However, based on the *R* value, the NARNET model has shown a better performance. In general, both models demonstrated an excellent prediction of the WQI values with *R*% > 93.93.

Figure 6 illustrate the histogram error of the NARNET model. The histogram metric is used to find errors between the target values and the predicted values of training and testing datasets. The total error range is divided into 20 smaller bins, where the *y*-axis refers to the number of samples located in a particular bin.  Figure 7 displays the histogram metric and mean errors of the LSTM model in the training and testing phases. The mean error and histogram metric are used to find the deviation between the observation values and the predicted values of training and testing.

Figures 8 and 9 display the regression plots for the predicted values of training, testing, and whole datasets for the NARNET and LSTM models, respectively. This plot is used to find the relationship between the predicted values and actual values. The “target” values in the plot are the actual dataset, whereas the “output” is the predicted values obtained from the NARNET and LSTM models. As shown in both figures, there is a clear good agreement (*R* > 95.7% (NARNET) and *R* > 93.3% (LSMT)) between the predicted WQI values and the ones calculated from the measured parameters. This implies the highly efficient performance of both developed models.

Table 7 summarizes the Pearson's correlation coefficient approach is used to predict the WQI values. The correlation between the WQI parameters for selecting the optimal parameters has been obtained. Results revealed that all parameters have a strong relationship with WQI parameters. This indicates that these parameters are very important for predicting the quality of water.

### 3.2. Prediction of the Water Quality Classification

This section presents the results of the classification algorithms are used to predict the WQC.  Table 8 shows the results of the used machine learning algorithms. It is noted that the performance of the SVM algorithm is very superior as compared to the KNN and Naive Bayes models. However, the Naive Bayes algorithm has shown the poorest performance.  Figure 10 shows the performance of the used algorithms to predict the WQC.

## 4. Conclusions

Modeling and prediction of water quality are very important for the protection of the environment. Developing a model by using advanced artificial intelligence algorithms can be used to measure the future water quality. In this proposed methodology, the advanced artificial intelligence algorithms, namely, NARNET and LSTM models were used to predict the WQI. Moreover, machine learning algorithms such as SVM, KNN, and Naive Bayes were used to classify the WQI data. The proposed models were evaluated and examined by some statistical parameters. For the WQI prediction, the result has revealed that the performance of the NARNET model is slightly better than the LSTM model based on the obtained *R* value. However, the SVM algorithm has achieved the highest accuracy of the prediction of the WQC as compared with KNN and Naive Bayes algorithms. After examining the robustness and efficiency of the proposed model for predicting the WQI, in future work, the developed models will be implemented to predict the water quality in Saudi Arabia for different types of water.

## Figures and Tables

**Figure 1:** Framework of the proposed methodology.

**Figure 2:** Computation of the NARNET model.

**Figure 3:** Architecture of the NARNET model.

**Figure 4:** Architecture of the DNN model.

**Figure 5:** Architecture of the LSTM model.

**Figure 6:** Histogram error of the NARNET model.

**Figure 7:** Histogram error and mean error of the LSTM model in the training and testing phases.

**Figure 8:** Regression plot of the NARNET model.

**Figure 9:** Regression plot of the LSTM model.

**Figure 10:** Performance of the machine learning algorithms used for the prediction of the WQC.

**Table 1:** Permissible limits of the parameters used in calculating WQI [43].

Parameters	Permissible limits
Dissolved oxygen, mg/l	10
pH	8.5
Conductivity, *μ*S/cm	1000
Biological oxygen demand, mg/l	5
Nitrate, mg/l	45
Fecal coliform, Cfu/100 ml	100
Total coliform, Cfu/100 ml	1000

**Table 2:** Parameter unit weights.

Parameter	Unit weight (*w*_*i*_)
Dissolved oxygen	0.2213
pH	0.2604
Conductivity	0.0022
Biological oxygen demand	0.4426
Nitrate	0.0492
Fecal coliform	0.0221
Total coliform	0.0022

**Table 3:** Water quality classification (WQC) [42].

Water quality index range	Classification
0-25	Excellent
26-50	Good
51-75	Poor
76-100	Very poor
Above 100	Unsuitable for drinking

**Table 4:** Parameters of the developed ANN (NARNET) model.

Number of hidden layers	12
Number of delays	1 : 8
Maximum number of iterations	100
Maximum number of epochs	12
Number of gradients	1.734 × 10^3^

**Table 5:** Parameters of the LSTM model.

Parameters	Numbers
Shallow hidden layer size	[30 80]
No. of hidden units 2	200
No. of hidden units 1	350
Delays	[1 3 4 7]
Maximum number of iterations	1500
Maximum number of epochs	150

**Table 6:** Performances of the NARNET LSTM and ANN models to predict WQI.

Models	Training data set			Testing data
	MSE	*R* (%)	MSE	*R* (%)
NARNET	0.2815	95.97	0.1353	96.17
LSTM	0.1316	93.93	0.1028	94.21

**Table 7:** Performance of Pearson's correlation coefficient approach.

Parameter	DO (mg/l)	pH	Conductivity (*μ*S/cm)	BOD (mg/l)	Nitrate (mg/l)	Fecal coliform (MPN/100 ml)	Total coliform (MPN/100 ml)	WQI
DO (mg/l)	1.00	0.0466	-0.2914	-0.1819	-0.0347	0.1128	-0.1536	-0.3836
pH	0.0466	1.00	0.3268	0.2697	0.0562	-0.2082	-0.2170	0.5233
Conductivity (*μ*S/cm)	-0.2914	0.3268	1.00	0.3288	0.1009	-0.1120	-0.0777	0.3935
BOD (mg/l)	-0.1819	0.2697	0.3288	1.00	0.2257	-0.1597	-0.1633	0.6130
Nitrate (mg/l)	-0.0347	0.0562	0.1009	0.2257	1.00	0.1408	0.0545	0.1768
Fecal coliform (MPN/100 ml)	-0.1128	-0.2082	-0.1120	-0.1597	0.1408	1.00	0.9119	0.2779
Total coliform (MPN/100 ml)	-0.1536	-0.2170	-0.0777	-0.1633	0.0545	0.9119	1.00	0.2679
WQI	-0.3836	0.5233	0.3935	0.6130	0.1768	0.2779	0.2679	1.00

**Table 8:** Performance of the used machine learning models to predict WQC.

Models	Accuracy (%)	Sensitivity (%)	Specificity (%)	Precision (%)	*F*-score (%)
SVM	97.01	99.23	97.78	94.93	98.54
KNN	83.63	84.73	94.93	87.50	85.84
Naive Bayes	75.20	77.76	91.65	78.08	81.51

## Data Availability

The dataset used in this study is collected from certain historical locations in India. It contained 1679 samples from different Indian states during the period from 2005 to 2014. The dataset has 7 significant parameters named dissolved oxygen (DO), pH, conductivity, biological oxygen demand (BOD), nitrate, fecal coliform, and total coliform. The data was collected by the Indian government to ensure the quality of the supplied drinking water. This dataset was obtained from Kaggle https://www.kaggle.com/anbarivan/indian-water-quality-data.
